# Sensory Integration Training and Social Sports Games Integrated Intervention for the Occupational Therapy of Children with Autism

This article has been retracted.

**DOI:** 10.1155/2022/9693648

**Published:** 2022-08-30

**Authors:** Zhen Wang, Yulong Gui, Wenwei Nie

**Affiliations:** ^1^Northeastern University, Shenyang Liaoning 110819, China; ^2^College of Physical Education, South-Central Minzu University, Wuhan Hubei 430079, China; ^3^Wuhan Yimixing Education Technology Co., Ltd., Wuhan Hubei 430000, China

## Abstract

This paper presents a research design for an integrated intervention using sensory integration training fused with social sports games for the treatment of children with autism. This study used a multiple baseline cross-subject design in a single-subject experiment, with structured play as the independent variable and expressive language skills of children with autism spectrum disorders as the dependent variable, with three phases of intervention: baseline, intervention period, and maintenance period. The expressive language ability was examined in terms of both oral expression and gestural expression, where the intervention effect of the oral expression was analyzed in terms of four components: the total number of words, the total number of sentences, average sentence length, and vocabulary complexity of oral expression, and the intervention effect of the gestural expression was analyzed in terms of changes in the frequency of children's gestural expression behaviors. For the categories classified by sensory integration ability, there are corresponding specific training programs that combine various physical exercises and play equipment to train the various abnormal functions of children with autism. Stereotyped behavior is a repetitive, self-imposed, and purposeless physical action, usually in the form of continuous and repetitive movements, sounds, and so on. 4 times a week, 25 minutes each time, the activity of recognizing pictures and familiar objects is carried out first, and then the children choose the structured game model and the initiative to build and take turns with the researchers to build. Stereotypic behaviors cause a great deal of distress in the lives of children with autism, and it is necessary to explore how to implement positive and effective interventions. Subjects' play abilities developed after receiving effective critical response training. The subjects' practice and symbolic play showed good immediate and maintenance intervention effectiveness; their associative and functional play showed no significant intervention effectiveness. The enhancement of the sensory integration skills of children with autism through sensory integration training resulted in a relative reduction of stereotypic behavior about the stimulus-seeking function, which had a positive effect on the intervention of stereotypic behavior.

## 1. Introduction

Among all types of special children, parents with children with autism experience greater stress and trials, which is one of the reasons why children with autism have always been in the limelight. The term autism first appeared as a medical term, and the concept of autism was first introduced in 1943 when Kanner named children with specific disorders that cause odd behavior problems as autistic children [1]. Researchers have not yet found a clear cause for autism, but as the number of children with autism increases, society is turning increased attention to this special group, and research on autism and its rehabilitation is becoming abundant. Not only do children with autism have serious problems of their own but they also have an indelible impact on their parents, who need to generate greater financial benefits to cope with the stress of treatment for their patients. Compared to the families of normal children, among the caregivers of children with autism, parents are in poorer health, have a more pessimistic psychological state, and have autism-like traits [2]. The main reasons for this situation are that autism is not easily accepted by society and peers, that autism requires long-term treatment, and that rehabilitation is expensive but treatment is weak, which can cause psychological depression in parents of children with autism, and long-term depression can affect all aspects of life, making parents more prone to anxiety and agitation, which, overall, causes a vicious circle. Therefore, we should not only focus on the physical treatment of children with autism but also on the psychological treatment of children with autism and their caregivers, which can be more helpful to the treatment of children with autism and can have twice the effect with half the effort.

The relationship between sensory integration disorder and stereotypic behavior has been discussed by scholars who are interested in this area because of the similarities in their behavioral manifestations and the confusion that can arise [3]. The main intrinsic reason for stereotypic behavior is to seek sensory stimulation. Because a large percentage of individuals with autism have sensory integration deficits and have difficulty maintaining a normal quiet state when given sensory stimulation, individuals with autism exhibit stereotypic behavior. Therefore, autistic individuals exhibit stereotypic behaviors to seek or avoid certain aspects of sensory stimulation. Later, some scholars further studied to elaborate the triggers of stereotypic or self-injurious behaviors in autistic individuals: to obtain or avoid sensory stimuli, to reach their homeostasis, and to regulate the sensory system. If the ability of autistic children to process sensory information can be made to improve, it is likely to improve their stereotypic behaviors [4]. Repeating the practice of the baseline period, the researchers played free games with the subjects, recorded the subjects' expressive language in the free games through video, and used language sample analysis tools to evaluate the subjects' expressive language changes. Based on this hypothesis, this study will attempt to use sensory integration training to improve the ability of children with autism to process sensory information about the external environment and investigate the effects of sensory integration training on improving stereotypical behaviors in children with autism. The theoretical implications of using structured games to intervene in the expressive language skills of children with autism are mainly in two aspects. First, there is a relative lack of theoretical results related to expressive language skills, and as an indispensable ability for children with autism to communicate and interact with peers and teachers, expressive language skills deserve further exploration by researchers; second, this study applies structured games to the expressive language skills of children with autism through a single-subject experimental method [5]. Second, this study applied structured games to children with autism to improve their expressive language skills through a single-subject experiment, which can provide empirical evidence to support the effectiveness of structured games in improving children's expressive language skills.

Play plays a critical role in children's development, promoting physical, cognitive, linguistic, social, emotional, and affective skills. Compared to normal children, children with autism have a deficit in symbolic play. These children tend to manipulate toys or objects rigidly or stereotypically and rarely initiate creative symbolic play activities spontaneously. Critical response training is an evidence-proven effective autism intervention that has demonstrated intervention effectiveness for a wide range of behaviors in children with autism. Intervention effectiveness, which can also be referred to as intervention validity, refers to the expected effects obtained from the study, including immediate and maintenance effects of the intervention. The immediate effect refers to the change of the participant during the intervention, the greater the change, the more significant the intervention effect; the maintenance effect refers to the maintenance time that the changed behavior can be maintained after the participant has completed all interventions: by screening the structured play model, developing a structured play intervention program, and using it in an intervention for expressive language skills of children with autism, to explore the effectiveness of structured play as an easy-to-implement, functional, and fun intervention that meets children with autism's preference for predictable, visualized objects to improve their expressive language skills. Based on the results of the study, appropriate recommendations are made to provide parents and teachers of children with autism concerning the teaching of expressive language to children with autism. Through the intervention of structured games, we help children establish a sense of rules of play and exercise their abilities in cooperation, fine and gross motor development, and joint attention.

## 2. Related Works

Spielmann and Porter found that children with autism often exhibit a range of low-motivation behaviors such as tantrums, disobedience, and inattention and attempts to escape the teaching environment [6]. Cahill et al. also found that lack of motivation is a common problem for children with autism and is what makes children with autism deficient in play and social interaction [7]. Other researchers have also found that the experience of completing tasks that are difficult or failing tends to make children with autism less motivated, which allows children to exhibit aggressive or disruptive behaviors. Therefore, some researchers have added motivational training to interventions in natural contexts to continuously increase the motivation of children with autism, resulting in not only effective improvements in children's abilities in areas such as play and language but also a reduction in their disruptive behaviors [8]. Self-management is the process by which individuals continuously plan and regulate their behavior actively and consciously to achieve predetermined goals [9]. Improving the self-management ability of children with autism allows them to learn to self-arrange and regulate themselves to better live, study, work independently, etc. In terms of communication, the main manifestation is the impairment of language development. Some children with autism have delayed or complete loss of verbal language development, those with some verbal ability have difficulty in using speech to communicate, and some children with autism have specific speech phenomena, such as echolalia.

In terms of social interaction, autistic children have a lack of nonverbal behaviors, such as eye contact, facial expressions, and body movements and a lack of interpersonal and emotional interactions. There is a lack of interpersonal and emotional interactions [10]. Since the kindergarten has a dance studio on the same floor, the teaching of sports games is carried out in indoor classrooms. There is an inability to actively share emotions such as joy with others; there is an inability to achieve the partnerships that children of the same biological age can establish. In terms of behavior patterns, they are compulsive, repetitive, and stereotypical [11]. Individuals with autism often focus wholeheartedly on one or more compulsive stereotypical and meaningless interest tendencies, such as compulsive attention to a certain type of shaped object; some individuals with autism often exhibit repetitive and stereotypical behaviors, such as biting fingers, walking in circles in place, and repeatedly kneading the corners of their clothes [12]. Beck et al. aimed to intervene in the social interactions of children with autism using peer-intervened critical response training [13]. Chung also found that peer-intervened critical response training had a very positive intervention effect on the social skills of children with autism during recess [14].

In summary, children's play abilities develop in a specific order, and research and interventions on children's play should be based on children's current play abilities and consider their developmental changes. In this study, according to the developmental order of children's playability, the main four levels of playability were classified as practice play, associative play, functional play, and symbolic play. Critical response training, as a natural intervention strategy, is based on the components of analogization and maintenance, which makes it easier for children to apply the acquired skills to natural situations and natural environments compared to other intervention strategies. Second, critical response training targets the “core domains” of children with autism, and once the intervention is effective, it is equally effective in other related domains, providing greater benefit to the child.

## 3. Sensory Integration Training Integrated with Social Sports Game Model Design

Sensory integration refers to the act of merging sensory information from various parts of the body's organs into one organization and then processing it by the brain to complete the perception of the inside and outside of the body and give feedback. With sensory integration, it is possible to ensure that the various components of the nervous system work together to make the individual engage with the environment smoothly. The theory states that the human body can respond to the environment because of sensory input, and that the integrative action of the brain can influence the form and degree of response. The development of the theory of sensory integration is based on the neurophysiology of the brain [15]. Its development follows the principles of brain and behavior development. Sensory integration can be simply understood as the process of inputting different sensory signals from the external environment to the brain, which processes the signals and makes appropriate responses. Humans can perform some daily, advanced, and complex behaviors and activities formally because they have undergone sensory integration. In plain language, sensory integration is a mutual learning process in which the human body and brain learn to harmonize with each other in response to the external environment. Without sensory integration, the human brain and body will not be able to develop and evolve. It is like the relationship between a traffic police officer and a traffic light. There are five main areas of sensory integration: vestibular ability, tactile ability, proprioception, learning ability, and special problems at older ages.

In human early childhood, sensory integration ability determines the strength of learning ability; so, if the development of sensory integration ability starts in early childhood, it will help the development of young children's psychological as well as emotional intelligence, but if the development of sensory integration ability is not coordinated, it will hinder the normal life and learning of young children. Therefore, we should pay attention to the development of the sensory integration ability of young children, and we should choose the appropriate sensory stimulation input for young children and combine it with body movement to lay a good physiological foundation for the development of young children's ability.

Children have strong plasticity in their nervous system during growth and development, and sensory integration training is to stimulate brain functions through training in auditory, visual, basic sensory, balance, and spatial perception, so that children can unify and merge these senses within themselves, and promote good physiological development of brain nerves and rational response, and its idea of changing behavior for the human brain behavior. The internal consistency of each dimension of the scale is 0.495-0.904, of which the alpha coefficients of social communication, social motivation, and autism behavior are all greater than 0.75, and the internal consistency is good. The total questionnaire is 0.954, indicating that the questionnaire has a good construct validity. In contrast, unlike sensory integration training, behaviorist therapy focuses on the relationship between behavior and environment and improves behavior by changing the environment, as shown in Figure 1.

Sensory integration refers to the physiological process by which the brain receives, processes, and feeds back various sensory information. An individual is considered to have a sensory integration disorder when his or her sensory integration ability is less than two standard deviations above that of his or her peers. Medical science classifies them into three main categories: sensory hypersensitivity, sensory retardation, and sensory stimulus seeking. Sensory hypersensitivity and sensory retardation are both caused by low or high response thresholds. Sensory stimulus seeking, on the other hand, is the excessive seeking of sensory experiences to satisfy sensory needs and is dangerous because of the inability to correctly anticipate the consequences of behavior due to intellectual disability.

Inclusive environments emphasize teachers creating cooperative situations, experiencing successful experiences gained through cooperation and negotiation in specific contexts, and providing opportunities to interact and engage with peers to promote the formation of a sense of cooperation in young children. Creating an inclusive environment is an effective prerequisite for cooperative learning between general peers and children with autism and can encourage reflection to reduce prejudice [16]. Creating an inclusive environment is an effective prerequisite for collaborative learning between regular peers and children with autism. Cooperative learning considered to have social advantages in inclusive school settings because it has been shown to increase the level of social participation of students with disabilities. Engaging students in the daily content of the classroom through natural support reduces differences through frequent use of relevant interpersonal and group skills. The presence of peers can increase the number and duration of social learning time. This is because there are more opportunities to communicate, observe others' behavior, initiate, share, imitate, collaborate, and solve problems.

The independent variable in this study was a structured game designed with Legos as the play material. Throughout the study, the researcher identified a total of 14 Lego models, including crocodiles, cameras, motorcycles, and castles, based on the developmental level of the three subjects. As the children mastered the skills, the researcher gradually increased the difficulty of the games. Each intervention was divided into three phases: preintervention, middle, and postintervention. In the preintervention phase, children first performed a picture recognition and familiarization activity, and then children chose the structured game model while choosing the initiative to build so that children understood and clarified the task of the model they were about to build; in the middle of the intervention, the researcher explained the building rules to children, children and the researcher each took turns to build 3 steps, and the researcher would give instructions to children during the game. The researcher would give instructions to the children, provide visual cues to assist children's expression, and set up sessions to stimulate children's spontaneous expression, such as giving one less or wrong block when it was the child's turn to play the role of the builder; the researcher could also set up sessions to build fewer blocks when he or she played the role of the builder [17]. It showed a downward trend in the late intervention period and maintenance period, and it was almost nonexistent in the end; its proper single-word initiation always showed a very low level, and there was no such initiation in the maintenance period. At the end of the intervention, the researcher asks the children three preset questions, summarizes with the children how they felt about building blocks, etc., and rewards the subjects with reinforcers according to their preferences.

In this stage, the researcher only plays freely with children without any special regulations on the game theme or game materials, which can be Lego or other neutral toys, and the teacher plays the game with children, who are free to choose toys and play with a certain kind of toy in the way they like, as shown in Figure 2.

This phase used structured games to intervene with the subjects sequentially, 4 times a week, 25 minutes each time, starting with a picture recognition and familiarization activity, and then the children chose the structured game model and the initiative to build and took turns to build with the researcher, who would give instructions to the children during the game, provide visual cues to assist children's expression, and set up sessions to stimulate children's spontaneous expression, such as the intervener building fewer blocks, MIS building blocks, and wrongly holding blocks. Reinforcers were given as rewards according to the subjects' preferences. After each intervention, the researcher played free to play with the subjects and video-recorded the children's expressive language performance during free play. 28 intervention sessions were given to each of the 3 subjects starting from week 2, week 3, and week 4, respectively.

One week after the end of the intervention period, the maintenance period was entered, and the researcher did not intervene with the subjects and repeated the baseline period. Five data points were collected for each of the three subjects. The proportion of children with BMI index in the obese and overweight range was 71.4%, and the proportion of children with BMI index in the mean range was 28.6%.

The experimental subjects were selected from children with mild autism who participated in the autism public service program; the children with autism who participated in the experiment were brought to the class by the autism public service organization, and the frequency of participation twice a week could be reliably guaranteed; the autistic children's rehabilitation association was not organizing other motor rehabilitation exercises during the period of participation in the experiment; the teachers who participated in this experimental program were all my colleagues [18]. The teachers who participated in this experimental program were all my colleagues, who were able to teach according to the designed curriculum, and all of them graduated from the physical education program and obtained the swimming instructor certificate.

Regular exercise is not only beneficial to the health of normal children but also has far-reaching implications for children with autism to improve their motor skills, increase their daily physical activity levels, and thus improve their physical health. Many researchers have also noted that exercise not only distracts and releases adverse emotions but also improves the individual's cognitive and language skills. Exercise as an intervention has been found to alleviate children with autism's symptoms, abnormal behaviors, and quality of survival 0. Therefore, ways to improve the physical fitness and illness of children with autism through exercise have also been noticed.

## 4. Occupational Experimental Design for Children with Autism

This study intends to make practical modifications to the theoretically constructed interactive physical activity program through the ascending logic of the action research cycle and finally form a practice-approved interactive physical activity intervention program for preschool children with autism. The kindergarten is new and has a small indoor space; so, the outdoor playground was chosen for physical play instruction. The classroom had only a few sets of toys, such as snowflakes, blocks, and plastic toys. Outside the classroom, there are small coasters, wooden horses, and other large toys; the kindergarten has a dance room on the same floor; so, physical education and games are taught in the indoor classroom. In addition to toys in the classrooms, the kindergartens have separate regional playrooms with recreational areas divided by function, such as a book area, a baking area, and a construction area [19]. Both kindergartens were equipped with complete sports equipment, such as basketballs, volleyballs, and other homemade play toys.

The whole study was divided into two phases: the baseline period and the intervention period. The content of physical games in both the baseline and intervention periods was appropriately adapted from the age-appropriate physical game curriculum of the middle school children, and all physical games were parallel games with no gradient changes. Coupled with the intense atmosphere of sports games, he took the initiative to cheer for other children, and the number of interactions with ordinary children also increased. There were 12 physical education game lessons, which were taught for 24 sessions of 25 minutes each, and each session consisted of 4 parts, as shown in Figure 3.

The entire experiment was conducted by three individuals: the researcher, teacher assistant A, and teacher assistant B. The researcher was responsible for teaching the experimental treatment period and administering all phases of the test uniformly; the teacher assistant was the observer and assisted the researcher in the physical education game intervention phase, and the entire process was videotaped.

The Social Responsiveness Scale is used to assess children's social skills and applies to children aged 4-18 years. It quantifies social skills and covers several aspects of behavior in social interactions, communication, and repetitive stereotyped behaviors in autism. The scale can be completed by a parent, another caregiver, or a teacher who knows the child's situation, based on the child's socialization with others in the natural environment over six months. The internal consistency of the scale was 0.495-0.904 for each dimension, with alpha coefficients greater than 0.75 for social communication, social motivation, and autistic behavioral styles, indicating good internal consistency, and 0.954 for the total questionnaire, indicating good construct validity.

The outline of the classroom teacher interviews was compiled by the researcher and was mainly used to understand the general teachers' knowledge about the situation of children with autism, the interaction between children with autism and general children in the school, and their views on the process and effectiveness of the physical education games incorporating cooperative learning strategies, to provide an empirical basis for the social validity analysis of the study. Parents of children with autism need to generate greater economic benefits to cope with the treatment pressures of their patients.

This phase of the physical game incorporating the independent variable cooperative learning strategy was designed with cross-subject multiple baselines; so, the cooperative learning strategy was added after the first group's baseline was stabilized, while the other groups of subjects remained at baseline. When the first group of dependent variables showed stable levels and trends, the independent variable was applied to the second group of subjects to implement the instructional intervention. When the second group of subjects showed stable levels and trends of the dependent variable, the independent variable applied to the third group of subjects, i.e., the experimental treatment period and the instructional intervention were implemented.

As shown in Table 1, the intervention period was identical to the baseline period in terms of session length and flow, with each session lasting 25 minutes and divided into 4 parts. The warm-up exercise in the first part and the game introduction in the second part used the same strategy, differing in the game in the third part and the closing activity in the fourth part. In the third part, 10 minutes of exercises and games are used. The intervention strategy uses the cooperative learning strategy until the end of the game. During the intervention period, the head teacher summarizes the performance of the students in the lesson and rewards the groups as well as individuals who have shown good cooperative learning.

The teacher selected this content for cooperative learning to be performed in the third part of the practice game and the formal game. The regular children worked with the autistic children on the physical education game tasks during the practice games and formal games. For example, when cooperative learning is not included, children with autism often practice alone [20]. Long-term depression will affect all aspects of life, making parents more prone to anxiety, excitement, and other emotions. If things go on like this, a vicious circle will result. When difficulties are encountered in the game, the teacher's assistance is part of the cooperative learning component, but what is deepened in this way is the emotional bond between the child with autism and the teacher. The interaction between regular and autistic children was facilitated by the fact that regular children played with autistic children in a negotiated and cooperative manner during practice play and formal play.

The rewards divided into material and social rewards. The material rewards were mainly stickers and candy. Social rewards were given along with material rewards to praise the children. For example, the researcher would first ask the group that showed the spirit of cooperation and helping each other to come up and then explain to the other children that their spirit of cooperation was shown by actively cooperating with their peers, completing the game successfully, and the following discipline. The first is to reinforce the groups that performed well to continue; the second is to encourage other children who did not perform well to learn from the groups that performed well.

## 5. Analysis of Results

### 5.1. Analysis of the Performance Results of the Integrated Intervention Model of Sensory Integration Training and Social Sports Games

The study used a self-initiation rating scale to observe the subjects' self-initiation, in which self-initiation was categorized as action-initiation, incomplete or inappropriate speech-initiation, appropriate single word-initiation, appropriate phrase initiation, and appropriate sentence initiation. A detailed analysis of the subjects' self-initiation was conducted, as shown in Figure 4. The subjects' action initiation was maintained at a certain level as the intervention progressed; their incomplete or inappropriate verbal initiation showed an increasing trend in the preintervention period and a decreasing trend in the postintervention and maintenance periods and was almost absent at the end; their appropriate single-word initiation remained at a very low level, and there was no such initiation in the maintenance period; their appropriate phrase initiation was relatively high in the baseline period and showed an increasing trend in the preintervention and maintenance periods. Subjects' appropriate sentence initiation also increased significantly after entering the intervention and showed an increasing trend in the maintenance period. Thus, it can be found that the subjects' lower levels of self-initiation decreased with the intervention, and their higher levels of effective initiation increased significantly with the intervention. Therefore, the results indicate that the critical response training has a good effect on the critical areas of the subjects, and it can effectively increase the high level and effective self-initiation of the subjects. People with autism appear to seek or avoid certain sensory stimuli through stereotyped behaviors.

Play is a very important learning opportunity for children, and thus, the development of play skills is crucial for achieving all aspects of children's development. The study analyzed the intervention effectiveness of critical response training on four play competencies: practice play, associative play, functional play, and symbolic play, respectively.

During the baseline period, the researcher administered four ratings to the subjects. All data points for this period distributed between 30% and 41.67%, with a mean value of 37.75%. There was an overall decreasing trend in the data during this period, with 3 points falling within the range of stability, which is 75%, meaning that there was a stable trend. Only one point in this period falls within the level range, and its level stability is 25%, indicating that this part of the data is unstable. However, statistical analysis of the data within the stage showed that *C* = 0.02, *Z* = 0.04, and *p* > 0.05, indicating that the variation in the rate of occurrence of habitual play behavior of the subjects within the stage was not significant.

During the intervention period, subjects received 16 ratings. The data points for this phase were distributed between 5% and 36.67%, with a mean value of 18.96%. The data in this phase also showed a decreasing trend, with 10 points falling within the trend stability range, with trend stability of 62.5%, indicating an unstable trend in the data. Only 6 data points fell within the level stability range in this period, with level stability of 37.5%, indicating that the data were also unstable. First, the theoretical achievements related to expressive language ability are relatively lacking, expressive language ability is an indispensable ability for autistic children to communicate and interact with their peers and teachers, and it is worthy of further research by researchers. The researcher used the *C*-statistic to statistically analyze the data within the intervention period, and the results were *C* = 0.47, *Z* = 2.01, *p* < 0.05, indicating a significant change in the rate of occurrence of the subjects' behaviors within the period; the interstage analysis of the data between the baseline period and the intervention period resulted in *C* = 0.66, *Z* = 3.10, *p* < 0.01, indicating that the subjects' practice play behaviors. There was an extremely significant difference in the rate of occurrence between the two phases; furthermore, the percentage of overlap between the two phases of data was 12.5%. The results of all analyses indicated that the subjects' rates of practice play behaviors decreased significantly after critical response training, showing a better immediate intervention effect.

A line graph was used to visualize the data on the subjects' practice play behaviors, where the horizontal coordinate is the number of evaluations and the vertical coordinate is the rate of practice play behaviors, as shown in Figure 5. The application of structured games to the intervention of autistic children's expressive language ability can provide empirical evidence for the effectiveness of structured games in improving the expressive language ability of autistic children. As can be seen from the figure, the percentage of the subjects' practice play behaviors in the baseline period was high, basically at 30% and above; after entering the intervention period, the percentage of the subjects' practice play behaviors tended to decrease, mostly at 25% and below; until the maintenance period, the percentage of the subjects' practice play behaviors continued to decrease, all less than 15%. Therefore, it can be tentatively determined that the critical response training has significant immediate and maintenance intervention effects on the subjects' practice play.

In addition, the percentage of overlap between the intervention period and the maintenance period data was 100%. The results of all analyses indicate that the rate of emergence of practice play behaviors decreased significantly after the subjects received critical response training, i.e., critical response training had a better maintenance effect on the subjects' practice play intervention. For example, when it is the child's turn to play the role of the builder, the researcher will give one less or the wrong piece of building blocks; the researcher can also set less building blocks when playing the role of the builder.

The initial dysregulation of sensory integration was severe, with severe dysregulation of tactile function, near-mild dysregulation of vestibular function, and moderate dysregulation of proprioceptive function. After three months of sensory integration training, there were significant improvements in all the functions of this case, among which the standard scores of tactile function and vestibular function increased by more than 15 points, and tactile function improved directly from severe to mild dysfunction, the vestibular function also improved to a large extent, and proprioceptive function improved from moderate dysfunction to mild dysfunction. From the results, the effect of sensory integration training on case C was obvious.

### 5.2. Analysis of Experimental Results

The social validity test of this training conducted mainly through interviews with the children's guardians, classroom teachers, and classroom teachers, and the training effect survey was conducted uniformly at the end of the study. After the interviews with the guardians, classroom teachers, and teachers were compiled, it was concluded that all of them felt that the three case children had improved after this training. Respondents felt that case A made significant progress in his emotional stability, motor volume, and motor coordination; case B made progress in gross motor, interaction with the outside world, and emotional control; and case C made progress in his tactile function and vestibular balance. 87.5% felt that case A had a better intervention effect, 62.5% felt that case B had a better intervention effect, and 75% felt that case C had a more effective intervention.

Case A's aunt felt that the child made significant progress, showed increased interest in movement, and had better intervention effects for behaviors such as finger wiggling, as well as increased positive emotions and better emotional stability. The brain processes the signals and responds appropriately. Humans can complete some daily, advanced, and complex behaviors and activities, which are officially considered as sensory integration. Case B's grandmother felt that her grandson had first improved in emotional control, several typical stereotypical behaviors had decreased, and he had improved in language. Case C's father felt that his son had less emotional control in the classroom, especially his irritability and tendency to lie down and cheat after a negative emotion, his motor activity had improved, and he had made progress in verbal communication and expression, as shown in Figure 6.

The height, weight, and BMI of the children with autism before the experiment and the changes in height, weight, and BMI of the children with autism after the experiment can be seen in Figure 6. After the experiment, 71.4% of the subjects had a decrease in BMI values greater than 0.5, 35.7% of the subjects had a decrease in BMI values greater than 1, and 7.1% of the subjects had a decrease in BMI values greater than 2 after the experiment.

Among the children with autism who had BMI tests before the experiment, the proportion of children with BMI in the range of obese and overweight was 71.4%, and the proportion of children with BMI in the range of mean value was 28.6%, and after the experiment, the proportion of children with BMI in the range of obese and overweight was 64.3%, a decrease of 7.1%. The proportion of children with BMI in the mean range after the experiment was 35.7%. Creating an inclusive environment is an effective prerequisite for collaborative learning with peers and children with autism that encourages reflection and reduces prejudice.

After 20 weeks of swimming practice, the children with autism had an improvement in their body shape or obesity and a decrease in their BMI, which is a very good sign for children with autism. It also indicates to some extent that swimming exercises can improve the body shape and body fat composition and obesity degree of autistic children to some extent and can play a certain effect on weight loss of autistic children.

According to the trend of change in inhibitory ability Figure 7, at the beginning of the experiment, the inhibitory ability of the control group was better, and after three months of intervention, the scores of the fourth measurement were the same, which shows that the trend and magnitude of improvement of the inhibitory ability of the experimental group were better than those of the control group.

Inhibitory ability refers to the ability to suppress dominant responses and respond to irrelevant stimuli during the performance of complex tasks. Creating an inclusive environment is an effective prerequisite for cooperative learning between ordinary peers and children with autism. A paired-samples *t*-test of the four measurements revealed that the experimental group showed significant differences between the four tests of inhibitory ability, while the control group showed significant differences between the tests except for the third month before and after the intervention. This indicates that interactive physical activities are more sustainable in improving the inhibitory abilities of preschoolers with autism compared to traditional physical education classes.

At first, the physical activity games did not appeal to him, but by the time the intervention expected, the regular children worked with him to complete the games, and with the intense atmosphere of the physical activity games, he took the initiative to start cheering for the other children and interacted more often with the regular children. He especially liked the part about choosing a companion, and sometimes, his eyes lit up when he heard that he had to choose a companion, and he also gave ideas when other children were choosing their companions.

## 6. Conclusion

Sensory integration training has a good practical significance in curriculum development and implementation, and the sensory integration training curriculum has good operability and feasibility and has a positive impact on children with autism. Sensory integration training has good curriculum validity and social validity, and it has a good effect on the improvement of children's sensory integration ability by setting the training contents for different children. Provide visual cues to assist children's expression and set up links to stimulate children's spontaneous expression. After enhancing the sensory integration ability of autistic children through sensory training, the stereotypical behavior of seeking a certain aspect of stimulation was also reduced, which had a positive effect on the intervention of stereotypical behavior. Critical response training was used to intervene in the critical areas of one child with autism to determine the effectiveness of critical response training intervention on the play abilities of children with autism. The subjects' practice plays and symbolic play showed better immediate intervention effectiveness and maintenance intervention effectiveness; their associative play and functional play had no significant intervention effectiveness. The structured play was effective in improving the expressive language skills of children with autism, and the immediate and maintenance effects of the intervention were positive. Structured games had better intervention effects on all dimensions of the expressive language ability of children with autism, and the intervention effect of the oral expression was better than that of the gestural expression.

## Figures and Tables

**Figure 1:** Sensory integration training framework.

**Figure 2:** Flow chart of social sports game intervention.

**Figure 3:** Course design.

**Figure 4:** Frequency of behaviors with different levels of self-initiation.

**Figure 5:** Rate of the emergence of play behaviors.

**Figure 6:** Statistics of height, weight, and BMI of children with autism before and after the experiment.

**Figure 7:** Intragroup comparison of inhibition ability in the experimental group.

**Table 1:** Intervention period physical education game lesson flow.

Teaching form	Duration	Content
Warm up	10 min	Regular roll call, low-intensity aerobic training
Game introduction	5 min	Explain the rules of the game
Game	15 min	Choose peers, cooperative learning
End event	5 min	Class summary and reward

## Data Availability

The data used to support the findings of this study are available from the corresponding author upon request.
